RETRACTED

# Biochanin A Gastroprotective Effects in Ethanol-Induced Gastric Mucosal Ulceration in Rats

**DOI:** 10.1371/journal.pone.0121529

**Published:** 2015-03-26

**Authors:** Maryam Hajrezaie, NurAin Salehen, Hamed Karimian, Maryam Zahedifard, Keivan Shams, Rami Al Batran, Nazia Abdul Majid, Shaden A. M. Khalifa, Hapipah Mohd Ali, Hesham El-Seedi, Mahmood Ameen Abdulla

**Affiliations:** 1 Department of Biomedical Science, Faculty of Medicine, University of Malaya, Kuala Lumpur, Malaysia; 2 Institute of Biological Sciences, Faculty of Science, University of Malaya, Kuala Lumpur, Malaysia; 3 Department of Experimental Hematology, Karolinska University Hospital, SE-141 86, Stockholm, Sweden; 4 Department of Chemistry, University of Malaya, Kuala Lumpur, Malaysia; 5 Division of Pharmacognosy, Department of Medicinal Chemistry, Uppsala University, SE-75 123, Uppsala, Sweden; University of California, Los Angeles, UNITED STATES

## Abstract

**Background:**

Biochanin A notable bioactive compound which is found in so many traditional medicinal plant. *In vivo* study was conducted to assess the protective effect of biochanin A on the gastric wall of Spraguedawley rats` stomachs.

**Methodology:**

The experimental set included different animal groups. Specifically, four groups with gastric mucosal lesions were receiving either a) Ulcer control group treated with absolute ethanol (5 ml/kg), b) 20 mg/kg of omeprazole as reference group, c) 25 of biochanin A, d) 50 mg/kg of biochanin A. Histopathological sectioning followed by immunohistochemistry staining were undertaken to evaluate the influence of the different treatments on gastric wall mucosal layer. The gastric secretions were collected in the form of homogenate and exposed to superoxide dismutase (SOD) and nitric oxide enzyme (NO) and the level of malondialdehyde (MDA) and protein content were measured. Ulceration and patchy haemorrhage were clearly observed by light microscopy. The morphology of the gastric wall as confirmed by immunohistochemistry and fluorescent microscopic observations, exhibited sever deformity with notable thickness, oedematous and complete loss of the mucosal coverage however the biochanin-pretreated animals, similar to the omeprazole-pretreated animals, showed less damage compared to the ulcer control group. Moreover, up-regulation of Hsp70 protein and down-regulation of Bax protein were detected in the biochanin A pre-treated groups and the gastric glandular mucosa was positively stained with Periodic Acid Schiff (PAS) staining and the Leucocytes infiltration was commonly seen. Biochanin A displayed a great increase in SOD and NO levels and decreased the release of MDA.

**Conclusions:**

This gastroprotective effect of biochanin A could be attributed to the enhancement of cellular metabolic cycles perceived as an increase in the SOD, NO activity, and decrease in the level of MDA, and also decrease in level of Bax expression and increase the Hsp70 expression level.

RETRACTED

## Introduction

Peptic ulcer is an open sore of resistant origin, provoked by multifactorial predispositions factors such as smoking, nutritional deficiency, stressful lifestyle, infections and frequent use of pain-killers such as nonsteroidal anti-inflammatory drugs (NSAIDs) [1,2]. Ulceration of the gastric wall is manifested by heartburn, nausea, stomach pain and discomfort and if not treated can lead to bleeding, perforation and loss of weight. The symptoms and discomfort accompanied with the gastric ulcer influence the quality of life and accordingly has social and economic implications [3,4]. The harmony between the immunological and hormonal systems assists the renewal of the gastric endogenous protective mechanism. A mechanism consisted of succession of events among them mucosal wall, blood flow, prostaglandins, epidermal growth factor, heat shock proteins, cathelicidins, lipoxins, nitric oxide and hydrogen sulfide [5]. Hydrochloric acid, pepsin and other chemicals irritate the lining of the stomach wall thus factors enhancing mucus production and/or suppressing stomach acid production can alleviate the pain and sooth the mucosal damage [6,3].

Antioxidants defend role against oxidative stress caused by necrotic agents is important factor to defend the gastric mucosa. Antioxidant can donate a hydrogen atom to reduce free radicals, preventing the process of lipid peroxidation by scavenging reactive oxygen species [1, 3]. Consequently finding new agents with safe effective mechanism that are possessing potent property and counteracting different etiological factors [7–9]. Medicinal plants are renewal source of new pharmaceutical leads. Natural products extracted from medicinal plants represent a new mean of alternative medicine to battle numerous illnesses [10–12] however further investigations are needed to prove their traditional uses. Habitual consumption of dietary flavonoids known to improve mitochondrial bioenergetics and inhibit various secondary outcome of reactive oxygen species (ROS) hence recommended as anticarcinogenic and chemopreventive possessions [13–15]. Biochanin A was characterized earlier as O-methylated isoflavone and a foremost aliment in soy and red clover [13]. Preclinical models suggest that flavonoids reduce gastric ulceration resulting from treatment with ethanol by opposing the excessive production of ROS [16], chelating metal ions and preventing lipid peroxidation [17]. There is considerable evidence supporting the harmful effect of Ethanol on gastric ulcers among others through oxidative stress and free radical theory [18]. As part of our ongoing projects to evaluate the biological activities of compounds extracted from medicinal plants and are currently commercially available, we attempt to investigate further the gastroprotective effect of biochanin A *in vivo*.

RETRACTED

## Materials and Methods

### Chemicals

Biochanin A was purchased from (Sigma-Aldrich. Com) and was dissolved in Tween 20 and given orally to rats at a dosage of 10mg/kg and 50mg/kg body weight (5 ml/kg). Omeprazole, reference antiulcer drug, was purchased from the Pharmacy of University of Malaya and was dissolved in the same amount and concentration of Tween 20 and administered orally at a dosage of 20 mg/kg body weight (5 ml/kg), as previously described by hajrezaie et al., 2012 [3].

### Ethical issues

This research protocol was permitted by the ethics committee for animal experimentation of the Faculty of Medicine, University of Malaya, Malaysia (Ethic No.PM/27/07/2010/MAA (R)) and the National Academy of Science’s Guide for the Care and Use of Laboratory Animals [19, 20].

### Experimental Animals

Healthy female adult *Sprague Dawley* rats (aged between 6–8 weeks and weighed between 200–220 g) were used. The animals were kept under standard laboratory circumstances, housed at temperature of 25 ± 2°C in a 12-hour light-dark cycle at the animal House Faculty of Medicine, University of Malaya, Kuala Lumpur, Malaysia. The rats were banned from any food, whilst had free access to water for 24 hours before treatment. Their admission to water was banned for 2 hours before the test started.

### Evaluation of acute toxicity

The acute toxicity study was carried out in adult female SD rats by the "fix dose" method of OECD (2002) (Organization for Economic Co-operation and Development) Guideline No.420 [20]. The procedure was implemented after dietary deprivation overnight with a starting dose of 250 mg/kg body weight. General, behavioural, neurological, and autonomic behaviour of the animal models were under observations during the experimental course [21].

### Induction of gastric ulcer

The rats were divided randomly into 4 groups, 6 animals each and the pretreatment was performed as previously described [3]. Group 1 (Ulcer control group, treated with absolute ethanol (5 ml/kg) base on the method recommended by Abdulla et al. [22], Group 2 (reference control group, feeding with 20 mg/kg omeprazole in 10% Tween 20 (5 mL/kg)). Group 3 and 4 (biochanin A with 25 and 50 mg/kg of 5 ml/kg), respectively. All rats were anesthesized by an overdose of xylazine and ketamine followed by cervical dislocation. The stomachs were dissected and put in normal saline.

RETRACTED

### Macroscopic examination of the gastric mucosal lesion

The length and width of the ulcer were measured with a planimeter (10 *×* 10 mm^2^) under a dissecting microscope (magnification: 1.8x). The ulcerated area was measured by calculating the total number of small squares underlying the ulcer band. The surface area of the lesions was then estimated as previously described [3], where “the sum of small squares ×4×1.8 = ulcer area UA (mm2)”. The inhibition percentage (*I* %) was calculated by the following formula:

$$\left(\text{I\%}\right)=\frac{\left(\text{UAcontrol}\;-\;\text{UAtreated}\right)}{\text{UAcontrol}}\times 100$$

### Detection of gastric wall mucus secretion

The gastric wall mucus was evaluated according to Corne et al. (1974) [23]. The glandular portion of stomach is weighed and transferred immediately to 10 ml of 0.1% w/v Alcian blue solution (0.16 M sucrose solution buffered with 0.5 ml of sodium acetate at pH 5). The tissue was kept in Alcian blue for 2 hours, and the excess colour was eliminated by consecutively rinsing it twice with 10 ml of 0.25 M sucrose. Dye combined with gastric wall mucus was extracted with 10 ml of 0.5 M magnesium chloride, which was irregularly shaken for 1 minute at 30-minute interval for 2 hours. Four millilitres of blue concentrate was then strongly shaken with an equivalent volume of diethyl ether. The achieved emulsion was spine at 3000 ×*g* for 10 minutes, and the absorbance of the fluid layer was recorded at 580 nm. The amount of Alcian blue concentrated for every gram of wet glandular tissue was afterwards calculated.

### Measurement of antioxidant and enzymatic activities

Superoxide dismutase (SOD) and nitric oxide (NO) levels were tested in the gastric tissue homogenate using the GSH and the SOD assay kits (Cayman Chemical Co., Mich, USA), following the manufacturer’s instructions. The gastric mucous membrane lipids peroxidation (MDA) was evaluated using the TBARS commercial kit (Cayman Chemical Co., Mich, USA).

### Measurement of protein concentration

Protein concentrations (mg/ml tissue) were measured using the Biuret reaction, as described earlier by Gornall et al. [24].

### Histological Studies of the Gastric Mucosa

#### Hematoxylin and Eosin

The stomach tissue of the different groups were fixed in 10% buffered formalin and sectioned by microtome (Leica, Germany). Sections of 5 mm thickness were then stained with hematoxylin and eosin.

#### Mucosal glycoproteins staining

Sections of the glandular layer within the gastric tissue were stained with PAS to differentiate the acidic and basic glycoproteins level in the mucus

RETRACTED

#### Immunohistochemical evaluation

Immunohistochemical staining was done according to standard protocol with few modifications (Dakocytoma- tion, USA). In Brief, the slides were heated for 25 min at 60C in a hot-air oven (Venticell, MMM, Einrichtungen, Germany), de-paraffinized in xylene and graded alcohol. Antigen retrieval was performed in 10 mM boiled sodium citrate buffer. Incubation with biotinylated primary antibodies namely Hsp70 (1:500) or Bax (1:200) was donefor 15 min followed by secondary labelling with streptavidin conjugated to horseradish peroxidase. Finally, counterstaining with DAB-substrate-chromagen was done prior to washing and hematoxylin addition.

### Statistical Analysis

The counts from different treatment groups were calculated from numerous microscopic observational fields and analysed for each individual experiment (n). Each experiment was repeated at least 3 times and triplicate samples were counted for each condition. Recorded data were fed into a computer program (Window XP, Excel). One-way ANOVA for independent samples with Tukey HSD as post hoc test was used for. A value of *P <* 0.05 was considered significant and all values were reported as mean *±* S.E.M.

## Results

### Evaluation of Toxicity

To evaluate the acute toxicity study, the rats were feed with the biochanin A bioactive compound for amount of 250 mg/kg and then were watched for two weeks. There was no sign of diarrhea, weakness, tremors, seizures or loss of controlled movement under the experimental period (Fig. 1). The effect of the plant extract on kidney and liver parameters like Chloride, CO2, Anion gap, Potassium, Sodium, Urea and Creatinine as renal parameters along with total protein, Albumin, Globuline, TB, CB, AP, GGT, AST and ALT as liver parameters in administered rats were considered and displayed no noticeable changes in comparison with control normal rats (Tables 1, 2).

**Fig 1:** Histological evaluation of acute toxicity assay. A and C) Control pre-treated with vehicle (10% Tween-20), B and D) pre-treated with 250 mg/kg of biochanin A. No structural differences were observed between the compound treated group and the control group. H & E stain; 100 x magnification.

**Table 1:** Effect of biochanin A on liver function biochemical parameters in rats.

Group	AST (U/L)	Albumin (g/L)	ALT (U/L)	T. Bilirubin (Umol/L)	AP (U/L)	T. Protein (g/L)
Vehicle 10% Tween 20	197.61 ± 27.06	41.14 ±13.17	47.75 ± 7.06	2.01 ± 0.57	148.03 ±23.14	55.24 ± 10.44
Biochanin A 250 mg/kg	183.08 ± 23.33	35.89 ± 9.79	40.87 ± 7.22	2.13 ± 1.60	137.97 ±21.55	48.71 ± 7.96

Values are expressed as the means ± S.E.M. There are no statistically significant differences between the measurements of different groups. Significance was set at *P* < 0.05.

RETRACTED

**Table 2:** Effect of biochanin A on renal function biochemical parameters in rats.

Group	Sodium (mmol/L)	Calcium (mmol/L)	Urea (mmol/L)	Potassium (mmol/L)	Creatinine (μmol/L)	Chloride (mmol/L)
Vehicle 10% Tween 20	163.22 ±14.25	2.27 ± 0.79	5.58 ± 1.28	5.76 ± 0.99	45.35 ± 7.38	114.57 ± 11.18
Biochanin A 5000 mg/kg	156.58 ± 5.13	2.10 ± 0.55	6.43 ± 1.14	5.63 ± 0.88	42.08 ± 5.13	110.95 ± 11.05

Values are expressed as the means ± S.E.M. There are no statistically significant differences between the measurements of different groups. Significance was set at *P* < 0.05.

### Macroscopic Evaluation of Gastric Lesions

Ulcers of the gastric mucosa appear as elongated bands of haemorrhagic lesions parallel to the long axis of the stomach. Gross evaluation of the dissected stomach (Fig. 2) showed clear damage to the mucosal capillaries and increased vascular permeability in the negative control group. On the contrast, biochanin A pre-treated group appeared typically healthy and viable. The surface area of the peptic ulcer zone is significantly small in biochanin A and positive control and the biochanin A interestingly made the gastric mucosal folds flattened compared to the untreated group (Table 3). The groups that treated with the biochanin A showed significant reductions in ulcer area (62.2%% and 74.68%; *p* < 0.05).

**Fig 2:** Macroscopical appearance of the gastric mucosa in rats. The negative control group (A) has no injury of gastric mucosa. The ulcer control group (B) displays sever injuries in the gastric mucosa. The reference control group (omeprazole, 20 mg/kg) (C) illustrations slight injuries in the gastric mucosa comparing to the injuries seen in ulcer control group. Rats fed with 25 (D) and 50 mg/kg (E) of the biochanin A has moderate injuries in the gastric mucosa.

**Table 3:** Effects of the biochanin A on gastric ulcer area, inhibition percentage and alcian blue binding capacity.

Animal’s group	pH	GWM (mg Alcian blue/g tissue)	Ulcer Area (mm)^2^	Inhibition (%)
Group1 (10%Tween 20) (ulcer control)	3.51 + ±0.04	130.05 ± 5.11	755.08 ± 20.17	-
Group 2 Omeprazole (20 mg/kg)	6.13 ±0.05*	621.18 ± 6.15*	172.45* ±19.22*	77.16%*
Group 3 Biochanin A (25 mg/kg)	4.88 ±0.04*	410.45 ± 5.22*	285.39 ± 6.86*	62.2%*
Group 4 Biochanin A (50 mg/kg)	5.78±0.06*	548.33 ± 4.16*	191.15 ±10.78*	74.68%*

Alcian blue binding capacity is defined as Gastric wall mucus (GWM).

Values expressed as mean ± S.E.M. There are no statistically significant differences between the measurements in different groups. The significant value was set at *P* < 0.05, compared with cancer control group.

RETRACTED

### Microscopic Evaluation of the gastric lesions

Based on the histopathological analysis, loss of the mucosal layer thickness was observed in the group treated with ethanol. On the other hand, biochanin A pre-treated group as well as positive control group showed better preservation of the gastric mucosa. The gastric tissues retain positive and uniform reactivity to the staining and the closely adherent mucosal layer contributed to the underlying cross-linking between biochanin A to the mucosal and glandular receptors. Biochanin A seemed to arrest the ulcerative processes which commence as soon as the mucosal layer is exposed to Ethanol. The assessment was done after the gastric luminal tissue has been processed, sectioned and stained to demonstrate the composition and appearance of tissue components (Fig. 3).

**Fig 3:** Analysis of Hematoxylin and eosin staining of the gastric mucosa. A) Gastric mucosa of the group exposed to ethanol. C) Gastric mucosa of the group treated with Omeprazole. C) Gastric mucosa of the group treated with 25 mg/kg biochanin A. D) Gastric mucosa of the group treated with 50 mg/kg biochanin A. The sections were cut parallel to the muscle layer. H & E staining, 100x magnification.

### Evaluation of Antioxidant and biochemical Activities

Tissue deprivation of the mucosal layer due to Ethanol treatment caused suppression of the NO, SOD expression, whereas in the group treated with biochanin A, the level of NO, SOD was interestingly high and presented a significant recompense surges (Table 4). Protein concentration was reduced where MDA level was increased in the homogenate extracted of the group treated with absolute ethanol. Usage of the biochanin A significantly increase the protein content and reduce the MDA proportion as illustrated in (Table 4).

**Table 4:** Effect of biochanin A on total protein concentration, antioxidant activity SOD, NO synthesis and level of MDA in gastric tissue homogenate.

Groups	SOD (U/mg protein)	NO (ng/mg protein)	MDA (μM/g protein)	Protein (mg/ml tissue)
Group1 (10%Tween 20) (ulcer control)	12.17 ± 0.31	1.52 + 0.001	212.61± 3.85	8.97 ± 0.33
Group 2 Omeprazole (20 mg/kg)	25.86 ± 0.35*	3.40 + 0.003*	131.23 ± 6.24*	14.06 ± 0.35*
Group 3 Biochanin A (25 mg/kg)	17.25 ± 0.26*	2.25 + 0.004*	164.25 ± 5.83*	11.58 ± 0.4*
Group 4 Biochanin A (50 mg/kg)	21.65 ± 0.42*	3.18 + 0.003*	139.81 ± 5.03*	13.25 ± 0.41*

All values are expressed as mean +- standard error mean. Mean difference is significant at the p<0.05 level and compared with cancer control group.

### Periodic Acid Schiff (PAS) staining

Upsurge in the glycoprotein content of the gastric mucosa was confirmed based on augment in the level of PAS staining in groups treated with biochanin A. The groups induced by ethanol showed the reduction in PAS staining level Fig. 4.

RETRACTED

**Fig 4:** Glycoprotein-PAS staining. A) Gastric mucosa of the group exposed to ethanol. C) Gastric mucosa of the group treated with Omeprazole. C) Gastric mucosa of the group treated with 25 mg/kg biochanin A. D) Gastric mucosa of the group treated with 50 mg/kg biochanin A. H & E staining, 100x magnification.

### Evaluation of immunohistochemical staining

Immunohistochemical outcome presented that animals in the groups 3–4 had high-regulation of Hsp70 protein. The expression of Hsp70 protein in groups treated with ethanol was down-regulated as compared to the group 3–4 (Fig. 5). Immunohistochemical analysis of Bax protein from the tissue section taken from groups 3–4 confirmed down- regulation of this protein. Administration of ethanol led to over-regulation of Bax, while fed with biochanin A reduced the appearance of this protein in the groups 3–4 (Fig. 6).

**Fig 5:** Immunohistochemical evaluation of the expression of HSP70 in the gastric tissues. A) Gastric mucosa of the group exposed to ethanol. C) Gastric mucosa of the group treated with Omeprazole. C) Gastric mucosa of the group treated with 25 mg/kg biochanin A. D) Gastric mucosa of the group treated with 50 mg/kg biochanin A. Immunohistochemical staining for HSP70 protein showed a up-regulation of HSP70 protein in the rats treated with the biochanin A. Magnification: 100x.

**Fig 6:** Immunohistochemical evaluation of the expression of BAX in the gastric tissues. A) Gastric mucosa of the group exposed to ethanol. C) Gastric mucosa of the group treated with Omeprazole. C) Gastric mucosa of the group treated with 25 mg/kg biochanin A. D) Gastric mucosa of the group treated with 50 mg/kg biochanin A. Immunohistochemical staining for HSP70 protein showed a down-regulation of BAX protein in the rats treated with the biochanin A. Magnification: 100x.

## Discussion

The acute toxicity experiment demonstrates no symbols of poisonousness or death in the practical amounts. Oral consumption of ethanol is harmful to the gastric organ which caused initiated regional disorder of gastric mucosa wall and stimulate outstanding alterations in vascular [25]. Absolute ethanol consumption formed haemorrhagic injuries, wide submucosal edema, mucosal frangibility, and damage to the epithelial cell of gastric tissue [26]. Secretion of mucus is supposed to be such as vital protective factor against gastric injuries. Ethanol would damage the mucosal layer as the important protecting layer of the gastrointestinal luminal cavity which banned straight interaction with the digestive enzymes [27]. Usage of ethanol led to decrease the protein concentration level followed by destruction of epithelial cells [28]. Omeprazole applied its function as a proton pump inhibitor and acid inhibitor agent which is offered equally protected role such as gastric mucosa, so in cure of sicknesses in relation with gastric acid secretion is widely used [29]. This agent is also effective as mucosal protection in treatment of non-acid depended models such as ethanol induced ulcer model [3, 7, 30].

RETRACTED

The results of the current research revealed that following fed the rats with biochanin A the protein concentration preserved in the homogenate stomach tissue. Treatment of the rats with biochanin A led to increase renewing of epithelial cells and so significantly augmented the protein concentration. Gastric motility is important in analysis of gastric mucosal damage /protection [31]. The more the folds are flatten the more the mucosal area are in contact with the agents [32]. In the current research one of the possible protective effect might be due to less of gastric motility. One of the protective way against harmful effect of ethanol on gastric mucosal is try to keep the normal level of nitric oxide to stop infiltration of the neutrophil [33]. Decrease in the level of nitric oxide NO and reduce the gastric blood flowing movement, following of that augment the level of Na+ and K+, producing pepsin as a result of consumption of ethanol, led to increase of lesions and so on caused the gastric mucus solubilised [33,34]. Based on the present study the biochanin A improved the activity of this enzyme which is in correlate with the pervious study [35].

Superoxide and hydroxyl radicals are main intermediaries of oxidative pressure that has important role in most of medical conditions. Thus, removing superoxide and hydroxyl radical has efficient effect to protect against disease [36]. The activity of SOD enzymes declines in response to the breakdown of the superoxide anion produced by lipid peroxidation. Decrease in the activity of SOD might lead to some harmful effects [37]. The group treated with the biochanin A revealed elevation in the activity of SOD whilst significantly decreased the level of malondialdehyde, as a sign for lipid peroxidation which get damage to cell membranes [38]. It is happened by an inaccuracy among oxidative injury and antioxidant protection systems. Decrease the level of lipid peroxidation after treated the rats with biochanin A resulted based on its antioxidant activity. Ethanol consumption led to morphologic alterations of gastric mucosa and made changes in biochemical parameters which are prevented significantly after treatment with biochanin A. MDA expression was significantly decreased in the group fed with biochanin A along with increased in SOD level.

RETRACTED

Based on previous studies the histological study of the gastric tissue presented that the features of ethanol-induced injuries contain inflammatory infiltrate, haemorrhage, edema, and loss of epithelial cells [39, 40]. The outcome result of the current research showed the defensive efficiency against gastric injury induced by ethanol following effect of biochanin A on banding leucocytes infiltration. Ethanol caused a notable reduction of the circular muscles which directed to mucosal density at the ridges of mucosal layers, which cause necrosis and ulceration [22]. The PAS staining technique displayed characteristic of stomach areas where the mucopolysaccharides is secreted [41]. This research revealed that the biochanin A improved gastric glands extreme mucus secretion. Apoptosis, programmed death of cells is able to activate by consumption of ethanol in the late phase of its infliction in the gastric epithelium. The increase level of Bax protein (proapoptotic factor) expression and decrease in the expression level of Bcl-2 (antiapoptotic factor) are two important sign of apoptosis pathway activation. Hsp70 protein, is highly expressed as a result of various types of stress. To keep the cellular homeostatic, it is vital to maintain the balance between the interaction among the proteins [42,43]. Ethanol let to produce reactive oxygen species which is prevent the expression of Hsp70 and upsurge Bax expression. The Hsp70 protein family play important role to deduct the intracellular denaturation of proteins induced by various stress issues. Besides of the chaperone activities, Hsp70 has been recommended to employ its gastro protective efficiency by mitochondria defensive role and by activation of apoptotic pathway [44]. The rats fed with biochanin A let to down regulation of Bax protein, which showed higher expression in the control group treated just with ethanol. Apoptotic cell death has significant effect to reduce the gastric mucosal entirety happened by numerous aggressive issues [44, 45]. Significant expression of Hsp70 as a gastro protective factor was initiate in the rats fed with biochanin A, brought this idea that the regulation of the proteins might has role in prevention of haemorrhagic mucosal injuries induced by ethanol consumption.

### Conclusions

Taken together, the regulation of the gastric cellular proteins noticed under biochanin A supplementation may play a role in prevention of mucosal haemorrhagic injuries and apoptotic programmed death induced by ethanol consumption. Biochanin A gastro protective efficiency can be claimed to the mitochondrial antioxidant cascade and activation of anti-apoptotic pathway.
